# Deep Learning-Based CT Imaging in Diagnosing Myeloma and Its Prognosis Evaluation

**DOI:** 10.1155/2021/5436793

**Published:** 2021-09-13

**Authors:** Jinzhou Wang, Xiangjun Shi, Xingchen Yao, Jie Ren, Xinru Du

**Affiliations:** ^1^Department of Orthopedics, Beijing Chaoyang Hospital, Capital Medical University, Chaoyang District, 100032 Beijing, China; ^2^Department of Hematology, Beijing Chaoyang Hospital, Capital Medical University, Chaoyang District, 100032 Beijing, China

## Abstract

Imaging examination plays an important role in the early diagnosis of myeloma. The study focused on the segmentation effects of deep learning-based models on CT images for myeloma, and the influence of different chemotherapy treatments on the prognosis of patients. Specifically, 186 patients with suspected myeloma were the research subjects. The U-Net model was adjusted to segment the CT images, and then, the Faster region convolutional neural network (RCNN) model was used to label the lesions. Patients were divided into bortezomib group (group 1, *n* = 128) and non-bortezomib group (group 2, *n* = 58). The biochemical indexes, blood routine indexes, and skeletal muscle of the two groups were compared before and after chemotherapy. The results showed that the improved U-Net model demonstrated good segmentation results, the Faster RCNN model can realize the labeling of the lesion area in the CT image, and the classification accuracy rate was as high as 99%. Compared with group 1, group 2 showed enlarged psoas major and erector spinae muscle after treatment and decreased bone marrow plasma cells content, blood M protein, urine 24 h light chain, pBNP, *ß*-2 microglobulin (*β*2MG), ALP, and white blood cell (WBC) levels (*P* < 0.05). In conclusion, deep learning is suggested in the segmentation and classification of CT images for myeloma, which can lift the detection accuracy. Two different chemotherapy regimens both improve the prognosis of patients, but the effects of non-bortezomib chemotherapy are better.

## 1. Introduction

Myeloma leads to increased levels of monoclonal immunoglobulin, which is attributed to malignant proliferation and abnormal accumulation of clonal plasma cells [1]. Studies have shown that the incidence of multiple myeloma has significantly exceeded that of acute leukemia and ranks second among hematological malignancies [2]. With the progress in research on treatment methods and the clinical promotion of hematopoietic stem cell transplantation technology, the complete remission rate of multiple myeloma has reached approximately 75% [3]. It has been confirmed that the median survival time of patients with multiple myeloma has been extended to 5 to 8 years [4]. Thanks to the unclear cause, the insidious onset, and low progress of myeloma, it is easy to cause the missed diagnosis and misdiagnosis [5]. In the treatment of myeloma, the chemotherapy regimen containing high-dose dexamethasone was generally selected in the past. This regimen has a rapid onset for newly discovered myeloma patients, with a median onset time of 1–1.5 months, which can quickly relieve patient symptoms. In recent years, with the emergence of new drugs such as immunomodulators and protease inhibitors, treatment programs have been further optimized. Nowadays, it is common to choose a combination of new drugs and traditional chemotherapy drugs for combined chemotherapy in clinical practice. This new combination chemotherapy regimen can significantly improve the remission rate of myeloma patients and the survival rate.

The clinical diagnosis method of myeloma is different from other general tumors. It requires obvious clinical symptoms of peripheral organ damage, such as renal function damage and osteolytic bone damage [6]. Recently, imaging techniques have been widely used in the diagnosis, differentiation, staging, and evaluation of therapeutic effects of multiple myeloma. Multiple myeloma is a blood system disease, involving multiple systems/organs. Systemic bone disease and extramedullary lesions have implications for the identification, diagnosis, and staging of the disease [7]. X-ray is always used in the imaging diagnosis of multiple myeloma, but it is positive only when more than 30% of the trabecular bone is destroyed and so it is easy to cause missed diagnosis [8]. CT imaging is characterized by cross-sectional scan, high-density resolution, and reconstruction. It is superior to X-ray scan in the diagnosis of multiple myeloma [9].

However, CT imaging cannot be used to stage the disease when there is no change in bone marrow infiltration and cortical bone. One of the most classic methods of deep learning is convolutional neural networks. Among them, Faster RCNN and U-Net are both earlier algorithms that use full convolutional networks for image segmentation. Deep learning used in the segmentation of medical images can greatly improve the segmentation effects [10]. The fully convolutional network (FCN) optimizes the fully connected layer in the traditional convolutional neural network into a convolutional layer, which reduces the complexity of the calculation and lifts the segmentation efficiency [11]. Compared with the FCN model, the U-Net model has higher segmentation accuracy and is not limited by the input sample size [12]. Using deep learning to process medical images can assist doctors in detecting lesions. It not only reduces the workload of doctors but also overcomes problems, such as poor diagnosis due to subjective differences.

In this study, a deep learning-based model was used to process CT images of patients with myeloma and then the effects of different chemotherapy treatments on the prognosis of patients were compared, aimed to provide reference for improving the clinical diagnosis, treatment, and staging effects of myeloma.

## 2. Methods

### 2.1. Research Subjects

A total of 186 suspected myeloma patients were selected, among whom 123 were initially diagnosed as myeloma by Durie–Salmon (DS) and International Staging System (ISS) methods. They all underwent surgery, pathological examination, and bone marrow aspiration biopsy and were diagnosed with myeloma. There were 93 males and 93 females, and the age ranged from 35 to 82 years, with an average age of 58.54 ± 10.15 years. The average interval between bone marrow biopsy and imaging examination was about 20 days.

The subjects were selected as per the following inclusion criteria: (i) those who met the diagnostic criteria for myeloma; (ii) those who had not received any radiotherapy, chemotherapy, or other therapies before treatment; (iii) those who had no other malignant tumors; and (iv) those agreeing with and accepting the study.

Exclusion criteria were as follows: (i) those with incomplete imaging data and (ii) those who cannot cooperate to complete the imaging examination. All patients have signed an informed consent form. All studies in this article have been approved by the Medical Ethics Committee.

### 2.2. CT Examination

The whole-body low-dose CT examination was performed using the Philips Brilliance ICT instrument. Under 120 kV and 50 mAs, the slice thickness was 2 mm, the slice spacing was 1 mm, the reconstruction slice thickness was 3 mm, the screw pitch was 0.811, and the collimation was 128 × 0.873 mm. During CT examination, the patient was in a supine position with arms crossed and placed on the lower abdomen. The scan was from the top of the skull to the proximal end of the tibia. After the scan, the collected images need to be transmitted to the image-processing workstation. The standardized bone algorithm was used to perform sagittal and coronal reconstruction.

### 2.3. CT Image Segmentation Based on U-Net

The U-Net model is used to segment skeletal CT images, and it is a typical “end-to-end” U-shaped network structure. To improve the segmentation effects, the original U-Net model was optimized, and the structure of the adjusted model is shown in Figure 1.

A loss function based on the Dice coefficient is used to balance the ratio of pixels in the bone area to the background area. The Dice coefficient is to measure the similarity between functions [13], and the Dice coefficient and its loss function are calculated as follows:

(1) $$\begin{array}{c} \text{Dice}=\frac{2\cdot \text{TP}}{2\cdot \text{TP}+\text{FP}+\text{FN}},\\ \text{loss}=1-\frac{2\cdot \text{TP}}{2\cdot \text{TP}+\text{FP}+\text{FN}}, \end{array}$$

TP is the number of positive samples predicted as positive samples, FP is the number of positive samples predicted as negative samples, and FN is the number of positive samples predicted as negative samples.

Intersection over union metric (IOU) is used to evaluate the segmentation effects. IOU calculates the intersection ratio, which is often used in the field of image segmentation [14]. The calculation of IOU is as follows:

(2) $$\begin{array}{c} \text{IOU}=\frac{\text{TP}}{\text{TP}+\text{FP}+\text{FN}}. \end{array}$$

### 2.4. Myeloma Detection Based on Faster RCNN

In order to realize the intelligent detection of myeloma using CT images, the Faster RCNN model is used to detect the lesion area. The Faster RCNN model mainly consists of two parts, namely, the region proposal network (RPN) and the region convolutional neural network (RCNN) [15]. The specific image processing steps using this model are as follows: First, the network classification model is used to extract the feature map, and then, the RPN is used to generate the region of interest (RoI), followed by the pooling operation. Finally, RCNN is used to classify the feature map and assign the probability value to the target category. The basic structure and parameters of Faster RCNN are shown in Figure 2.

The VGG basic model is used to extract the feature map. The basic structure of the VGG model is shown in Figure 3. The convolutional kernel sizes in the VGG model are 1 × 1 and 3 × 3. The activation function is a softmax function, and the reshape operation is performed before and after treatment to improve the classification effects.

The sample is input into the model for training, and the loss function of the model needs to include the RPN and detector, but the loss function is composed of classification loss and regression loss function, expressed as follows:

(3) $$\begin{array}{c} L\left(\left\{p_{i}\right\},\left\{t_{i}\right\}\right)=\frac{1}{N_{c}}\sum L_{c}\left(p_{i},p_{i}^{*}\right)+\alpha \frac{1}{N_{r}}\sum p_{i}^{*}L_{r}\left(t_{i},t_{i}^{*}\right), \end{array}$$

where *p*_*i*_ is the probability of the target area in the prediction box and *p*_*i*_^*∗*^ is the multiclass labels in softmax regression.

The mathematical expressions of classification loss *L*_*c*_ and regression loss *L*_*r*_ are as follows:

(4) $$\begin{array}{c} L_{c}\left(p_{i},p_{i}^{*}\right)=-\log\left(p_{i}^{*}p_{i}+\left(1-p_{i}^{*}\right)\left(1-p_{i}\right)\right),\\ L_{r}\left(t_{i},t_{i}^{*}\right)=R\left(t_{i},t_{i}^{*}\right), \end{array}$$

where *R* is the smooth *L*1 function, *t*_*i*_ is the offset of the prediction frame during the RPN training process, and *t*_*i*_^*∗*^ has the same dimension as *t*_*i*_. With the iteration of the loss function, the parameters of the softmax classifier are further optimized and clarified, which can distinguish different training samples.

### 2.5. Remission Induction Treatment Plan

With patients' economic levels and clinical differences taken into account, there were mainly two treatment plans: group 1 underwent bortezomib treatment, and group 2 underwent non-bortezomib treatment. There were 128 patients in group 1, and 58 patients in group 2.

### 2.6. Evaluation and Follow-Up

All patients were tested for laboratory indicators before treatment and after induction treatment, including blood routine, serum/urine protein electrophoresis, biochemical items (albumin, globulin, and blood creatinine), urine routine, and bone marrow examination, to explore clinical efficacy. All patients were followed up from the first visit, and the follow-up time was approximately 40 months. The overall survival time in this study was from the time of diagnosis to the end of the last follow-up. When patients were transferred halfway or gave up treatment, they were not included in the study of overall survival.

### 2.7. Statistical Processing

SPSS19.0 was used to process the data. Measurement data conforming to normal distribution were expressed as mean ± standard deviation, and comparisons between groups adopted the independent sample *t* test; measurement data that did not conform to normal distribution were represented by the median value, and the nonparametric rank sum test was used to analyze the difference between groups. The count data were expressed by percentage *n*, and the *χ*^2^ test was for comparison between groups. *P* < 0.05 was the threshold for significance.

## 3. Results

### 3.1. Segmentation Performance of the U-Net Model

U-Net and the improved U-Net′ network were trained for 50 rounds, and the loss curve and IOU curve of the two models on the training set and the test set were compared before and after chemotherapy. It is noted in Figure 4 that the loss curve of the U-Net′ model on the training set and the test set converged more quickly, while the area under the IOU curve was larger.

The loss value and IOU value were compared between the U-Net and U-Net′ model when the maximum training times are reached, and the results are shown in Figure 5. It was noted that the loss values of the U-Net′ model on the training set and the test set were larger, than the IOU value.

Subjectively, the segmentation effects of the U-Net and U-Net′ model on CT images were compared for multiple myeloma, and the results are shown in Figure 6. The segmentation effects of the lesion area on the T1 and T2 images were compared. It was noted that the U-Net model had poor effects when segmenting small lesions in the CT image and the improved U-Net′ model can realize the segmentation of small lesions. The red area in the figure is the segmentation of the lesions of myeloma patients under the U-Net model algorithm.

### 3.2. Detection and Verification of the Faster RCNN Model

The Faster RCNN model was trained, and the training results are shown in Figure 7. It was noted that when training iterations were below 10 times, the classification accuracy and loss value of the model gradually stabilized. The classification accuracy of the Faster RCNN model was approximately 0.966, and the loss value was approximately 0.092.

The trained Faster RCNN model was then used to detect multiple myeloma, and the results are shown in Figure 8. It was noted that the classification results displayed the prediction frame, the corresponding category, and the probability value of the target area. The red area in the figure is the part of the myeloma patient's lesion that was separated under the Faster RCNN model algorithm.

### 3.3. Basic Information of Patients

The baseline data of patients in group 1 and group 2 were compared, and the results are shown in Table 1. It was noted that there was no statistically significant difference between the two groups of patients in age, height, weight, gender, DS staging, and ISS staging (*P* > 0.05). Hence, the baseline data of the two groups were comparable.

### 3.4. CT Imaging for Waist Muscle of the Patient before and after Chemotherapy

The fat in psoas major, quadratus lumborum, erector spinae, and erector spinae was compared before and after chemotherapy, and the results are shown in Figure 9. It was noted that in group 2, the quadratus lumborum muscle was significantly reduced and the erector spinae muscle was significantly enlarged after treatment (*P* < 0.05) compared to before treatment; the psoas major and erector spinae muscle were significantly enlarged after treatment in group 2 compared to group 1, and the erector spinae muscle fat was significantly reduced (*P* < 0.05).

### 3.5. Biochemical Indicators before and after Chemotherapy

The ratio of bone marrow plasma cells, monoclonal immunoglobulin (M protein), urine 24 h light chain, pBNP, and *ß*-2 microglobulin (*β*2MG) levels were compared before and after chemotherapy, and the results are shown in Figure 10. It was noted that compared to before treatment, the levels of urine 24 h light chain, pBNP, and *β*2MG in group 2 were significantly reduced (*P* < 0.05) while the level of *β*2MG in group 1 was also significantly reduced (*P* < 0.05). Compared with group 1, the ratio of bone marrow plasma cells, blood M protein, urine 24 h light chain, pBNP, and *β*2MG levels were significantly reduced after treatment in group 2 (*P* < 0.05).

### 3.6. Blood Routine Indexes before and after Chemotherapy

The blood routine indexes of ALP, LDH, Cr, Alb, Ca, WBC, Hb, and Plt were compared before and after chemotherapy, and the results are shown in Figure 11. It was noted that compared with before treatment, the Cr levels of group 1 and group 2 were significantly reduced (*P* < 0.05). Compared with group 1, ALP before and after treatment in group 2 was significantly lower (*P* < 0.05), the LDH level before and after treatment was significantly higher (*P* < 0.05), and the WBC level after treatment was significantly lower (*P* < 0.05).

## 4. Discussion

Threshold segmentation is the most common image segmentation method. The pixel values in the target area and background are similar, but the pixel values of different target areas are different. The algorithm segments the target area according to the peak value displayed in the histogram [16]. Traditional segmentation algorithms are affected by image noise and other factors, and thus, they tend to have poor segmentation results. The U-Net model has been proved to have excellent segmentation results [17], so it was used in the study. Its parameters were adjusted based on the original one, and then, the adjusted one was used to segment the lesion area in CT images. It was found that compared to the original one, the improved U-Net model demonstrated better convergence effects and the area under the IOU curve was larger. It suggested that the adjusted U-Net model had better segmentation effects on the CT image of multiple myeloma. Image processing is an integral part in the detection of lesion area [18]. The deep learning-based model needs to classify the target areas after the recognition and positioning [19]. Therefore, the Faster RCNN framework was used to detect the lesion area on CT images for myeloma and to locate the target area in the CT image and label the category. The results showed that the Faster RCNN model can realize the positioning and category labeling of the lesion area, which lifted the diagnosis efficiency.

Plasma cells are transformed into protoplasmic cells by B lymphocytes after antigen stimulation, and protoplasmic cells evolve into mature plasma cells through processes such as differentiation and reproduction [20]. M protein is an abnormal immunoglobulin produced by the monoclonal malignant proliferation of plasma cells or B lymphocytes [21]. Studies have confirmed that the proportion of plasma cells and the level of M protein in patients with multiple myeloma are significantly increased [22]. The results of this study found that the proportion of bone marrow plasma cells and the level of M protein in patients undergoing chemotherapy were significantly reduced and the decrease in the non-bortezomib group was more obvious. The molecular structure of immunoglobulin can be divided into two types: heavy chain and light chain, of which the light chain is divided into *κ* type and *λ* type [23]. The multiple myeloma arises from excessive proliferation of abnormal plasma cells in the bone marrow, which in turn causes an increased level of M protein, lifting the level of urinary light chains, so the level of light-chain type of urine protein is an indicator for the diagnosis of multiple myeloma [24, 25]. *β*2MG is a small molecular protein synthesized by lymphocytes, which can be used to assess kidney function and can also be used for auxiliary diagnosis of malignant tumors [26, 27]. It was found in the study that, after non-bortezomib treatment, the patients' urine 24 h light chain and *β*2MG levels were significantly reduced, indicating that the treatment can effectively improve the prognosis of patients.

## 5. Conclusion

The purpose of this article is to use deep learning technology to segment and classify myeloma CT images and to further improve the clinical diagnosis and treatment of myeloma patients. The results showed that U-Net and Faster RCNN models can realize lesion area segmentation and labeling. The effects of different chemotherapy treatments on the prognosis of patients were compared. It was found that non-bortezomib treatment can significantly reduce the proportion of bone marrow plasma cells, M protein, urine 24 h light chain, *β*2MG, and WBC levels, indicating that the treatment plan can improve the patient's chemotherapy effects. However, some limitations in the study should be noted. The deep learning is only used to segment and classify the lesion area in the CT image and not applied to the CT image after chemotherapy. However, the research content of this article still has certain limitations. The article does not analyze the correlation between different prognostic indicators and the overall survival of patients. And, this article only studies a single imaging diagnostic method, so more imaging diagnostic methods will be studied in depth in the future. Therefore, more clinical indicators will be involved in the follow-up, to strengthen the findings of the study. In summary, the results of this study can effectively improve the diagnostic accuracy of patients with myeloma, provide certain guidance for subsequent clinical treatment, and significantly improve the prognosis of patients. It provides a certain theoretical basis for the subsequent research on imaging examination methods.

## Figures and Tables

**Figure 1:** Basic framework and parameter settings of the U-Net model.

**Figure 2:** Basic structure of Faster RCNN.

**Figure 3:** Basic structure of the VGG model.

**Figure 4:** Loss and IOU curves on the training set and test set.

**Figure 5:** Loss and IOU values on the training set and test set.

**Figure 6:** Segmentation of CT images for multiple myeloma.

**Figure 7:** Classification accuracy and loss curve of the Faster RCNN model.

**Figure 8:** The detection results of the Faster RCNN model for multiple myeloma.

**Figure 9:** CT results of the patient's psoas major before and after chemotherapy. The four pictures show (a) psoas major, (b) quadratus lumborum, (c) erector spinae, and (d) erector spinae fat. Compared to before treatment, ^#^*P* < 0.05; compared to group 1, ^*∗*^*P* < 0.05.

**Figure 10:** Biochemical indicators of the patient before and after chemotherapy. The five pictures show (a) bone marrow plasma cell ratio, (b) blood M protein, (c) urine 24 h light chain, (d) pBNP, and (e) *β*2MG. Compared to before treatment, ^#^*P* < 0.05; compared to group 1, ^*∗*^*P* < 0.05.

**Figure 11:** Routine blood indicators of patients before and after chemotherapy. The eight pictures were ALP, LDH, Cr, Alb, Ca, WBC, Hb, and Plt. Compared to before treatment, ^#^*P* < 0.05; compared to group 1, ^*∗*^*P* < 0.05.

**Table 1:** Comparison of baseline data between the two groups.

Project		Group 1 (*n* = 128)	Group 2 (*n* = 58)	Statistics	*P*
Age (year)		58.93 ± 9.65	57.69 ± 11.12	*t* = 0.771	0.441
Height (m)		1.66 ± 0.08	1.65 ± 0.10	*t* = 0.453	0.652
Weight (kg)		67.52 ± 10.51	66.85 ± 11.86	*t* = 0.317	0.752
Gender (*n*/%)	Male	69/53.91	24/41.38	*χ*^2^ = 0.839	0.334
	Female	59/46.09	34/58.62		
DS staging (*n*/%)	I	3/2.34	4/6.90	*χ*^2^ = 0.873	0.467
	II	9/7.03	4/6.90		
	III	2/1.56	1/1.72		
	IV	9372.66	39/67.24		
	V	20/15.63	9/15.52		
ISS staging (*n*/%)	I	17/13.28	10/17.24	*χ*^2^ = 0.797	0.562
	II	54/42.19	22/37.93		
	III	52/40.63	22/37.93		
	IV	0/0.00	0/0.00		
	V	1/0.78	0/0.00		

## Data Availability

The data used to support the findings of this study are available from the corresponding author upon request.
